The article "Investigation on Quality of Life and Economic Burden of Children with Cerebral Palsy in Changzhou" was retracted in 2023. Reasons: suspected computer-generated content; unreliable results or conclusions; concerns about the data; concerns about the results or conclusions.

# Investigation on Quality of Life and Economic Burden of Children with Cerebral Palsy in Changzhou

**DOI:** 10.1155/2022/1519689

**Published:** 2022-01-04

**Authors:** Chaorong Bian, Feng Peng, Haibin Guo, Kejin Chen

**Affiliations:** ^1^Changzhou Children's Hospital Affiliated to Nantong University, Changzhou 226019, Jiangsu, China; ^2^Changzhou Maternal and Child Health Care Hospital, Changzhou 213000, Jiangsu, China

## Abstract

Based on the data of children with cerebral palsy (CP) in Changzhou obtained by the Disabled Persons' Federation, this study sampled some children with CP and investigated their survival status, treatment cost, and family burden so as to provide scientific decision-making basis and policy suggestions for coping with disease hazards and improving children's quality of life. In this study, a simple random sampling method was used to conduct household surveys of the selected children with CP. The economic burden of CP is measured by direct and indirect methods, and the quality of life of patients of children with CP and their families is analyzed qualitatively and quantitatively by the EuroQol Five Dimensions (EQ-5D) Questionnaire. The average family economic burden of each case of CP in Changzhou was about 4,188,500 yuan, of which the direct medical burden was 205,800 yuan and the indirect economic burden was 3,982,700 yuan. The socioeconomic burden of CP in Changzhou is as high as about 2.244 billion yuan. From the EQ-5D measurement results of 55 children with CP, the average index score was 0.423, which was lower than the national general population level. The proportions of patients with CP who have problems in the five aspects of action, self-care, daily activities, pain/discomfort, and anxiety/depression are 72.73%, 81.82%, 81.82%, 83.64%, and 92.73%, respectively, which are significantly higher than those of the national general population. The average score of the Visual Analogue Scale (VAS) is 58.09, which is significantly lower than the national general population level. The only major factor affecting the quality of life of patients with CP and their families is the health status represented by the EQ-5D score. To liberate and develop the labor ability of patients and their direct caregivers through clinical treatment, rehabilitation, and special education is the most effective way to reduce the socioeconomic burden of CP. Relevant government departments should perform their duties, integrate social assistance resources, implement early intervention, and launch targeted support and assistance policy.

## 1. Background

Cerebral palsy (CP) in children has become the most serious disease problem affecting children's health worldwide. The incidence of CP in China is about 2.48% [1]. Based on a population of 12 million born in 2020 [2], there were approximately 29,760 children with CP born in China. Cerebral palsy patients are mainly manifested as dyskinesia and abnormal posture, accompanied by mental retardation, epilepsy, sensory disturbance, language disorder, and abnormal mental behavior. CP not only has an irreversible impact on the health of patients but also seriously affects their quality of life. In the meantime, it also brings a heavy economic burden to society and families, causing a series of social problems.

The article "Investigation on Quality of Life and Economic Burden of Children with Cerebral Palsy in Changzhou" was retracted in 2023. Reasons: suspected computer-generated content; unreliable results or conclusions; concerns about the data; concerns about the results or conclusions.

In terms of physical function, patients with CP have poor normal mobility and self-care ability, and most of them cannot take care of themselves. From the point of view of emotional function, they are emotionally unstable and vulnerable, and they are prone to fear, depression, anxiety, and other negative emotions. As far as social interaction, they rarely communicate with other children normally and lack corresponding entertainment activities. The total scores of children with CP in the Pediatric Quality of Life Inventory Measurement Models (PedsQL™) are lower than those in the normal control group or the general disease group [3]. Therefore, the training they usually have to receive includes big motor training, fine motor training, language cognitive training, life self-care ability training, and sensory integration training.

The economic burden of CP includes direct medical expenses, rehabilitation costs, long-term care costs, special education, and other expenses, as well as indirect loss of their productivity and the parents' income. The cost of the disease is an “opportunity cost” that reflects the burden of disease on society. If the disease can be reduced or even eliminated, society can reduce the cost of the disease and thus obtain benefits [4]. At present, research on the economic burden of CP is mainly concentrated in developed countries with abundant data resources and relatively prominent birth defects. The Nordic countries are known for their strong welfare systems, yet it is unknown to what extent the added burden related to disability is actually compensated for [5]. In Canada, direct health care costs in constant 2010 Canadian dollars were about $11,700 for children with cerebral palsy aged 1–4 years versus about $600 for those without the condition [6]. China has less research literature on this. Searching for “cerebral palsy” and “disease burden,” “economic burden,” “costs,” and “economic evaluation,” respectively, as keywords, there are fewer documents. Part of the literature only briefly describes the family economic burden of children with CP, which is not conducive to the government and society to provide targeted support and assistance, especially in Jiangsu Province, which accounts for 6% of the Chinese population [7]. Therefore, this study is based on the data obtained by Disabled Persons' Federation for children with CP in Changzhou, Jiangsu Province. We did a random sample and then investigated the quality of life and economic burden of those children to evaluate and analyze the related issues caused by CP from multiple perspectives such as society, family, and intervention.

The article "Investigation on Quality of Life and Economic Burden of Children with Cerebral Palsy in Changzhou" was retracted in 2023. Reasons: suspected computer-generated content; unreliable results or conclusions; concerns about the data; concerns about the results or conclusions.

Theoretically, the total economic burden of disease should be composed of direct economic burden, indirect economic burden, and intangible economic burden. We plan to use quantitative and qualitative analysis methods for evaluation. Among them, the direct and indirect economic burdens, such as the expenses invested by the family of children with CP, the time consumed, and the items purchased, can be directly obtained through questionnaire surveys, then calculated through quantitative analysis methods and mathematical formulas, and expressed in the form of monetary amounts. Limited by actual conditions, the actual number of patients receiving treatment is generally less than the number of illnesses or patients, so the direct economic burden of the disease will be overestimated by the direct method. In order to avoid overestimation, it is necessary to comprehensively consider the utilization rate of receiving medical services. We have taken this into consideration when calculating the economic burden of children with CP in Changzhou. The intangible burden is mainly qualitatively evaluated through interviews, which can understand the main problems, practical difficulties, ideological concerns, mental pressure, and needs of patients and their families.

The economic burden of CP is very sensitive to many objective factors such as China's regional socioeconomic development, family economic conditions, parents' educational level, disease severity, and treatment and rehabilitation methods, so in fact, the family economic burden of patients varies greatly. It is more difficult to calculate the economic burden. The direct economic burden of most surviving patients with birth defects is relatively small, and the indirect and intangible burdens are relatively large. This calculation requires more data sources, which greatly limits the estimation of the economic burden. Although the current research on the economic burden of CP has obtained some meaningful results, our research can provide the possibility of further improvement.

## 2. Materials and Methods

### 2.1. Survey Object

The inclusion criteria of the study objects are children under 14 years of age who have lived in Changzhou for more than one year with a clear diagnosis of cerebral palsy. Using the random number table method, a random sampling was carried out from 220 children with confirmed CP under 14 years old in Changzhou. The 55 selected children with CP were investigated one by one. Randomly selected children and their caregivers (parents, grandparents, etc.) were the respondents of this survey.

The article "Investigation on Quality of Life and Economic Burden of Children with Cerebral Palsy in Changzhou" was retracted in 2023. Reasons: suspected computer-generated content; unreliable results or conclusions; concerns about the data; concerns about the results or conclusions.

### 2.2. Survey Content and Methods

The questionnaire used in this survey has been used in the investigation of children with CP in Hebei Province in China [8]. The questionnaire contains five parts: sociodemographic characteristics, direct economic burden, indirect economic burden, daily activity ability, and quality of life of children with CP and their families (see Appendix 1). The questionnaire has been verified to have high reliability and validity. The measurement and evaluation methods of quality of life and economic burden are scientific and rigorous (see Appendix 2).

The investigator used a household survey to interview each child with CP and his family's direct caregiver and filled out questionnaires. The survey was jointly completed by children follow-up personnel and researchers in the area where the samples were located.

### 2.3. Statistical Analysis Methods

All questionnaires and content items are uniformly coded and entered by EpiData (Version 3.1). After checking the errors of the input data manually and computer logic, the conversion is performed, and SAS (Version 9.3) is used for statistics and analysis. If the measurement data obey a normal distribution, the discrete trend is expressed by the mean plus and minus the standard deviation; otherwise, the median (lower quartile; upper quartile) is used to express. The classification data is described by rate or composition ratio. The correlation of the quality of life of children with CP and their families was analyzed by the Spearman rank correlation analysis. The factors affecting the quality of family life were analyzed by logistic regression, with the inclusion criteria *α* = 0.05 and the exclusion criteria *α* = 0.10.

### 2.4. Investigation Quality Control

We conducted unified training for investigators participating in household surveys to clarify the purpose of the investigation, the investigation discipline, the tasks, and the requirements of the investigators and to be familiar with the investigation items. At the same time, the relevant knowledge of birth defect diseases, quality of life, and disease economic burden was briefly introduced.

Make sure that the investigator visits the families with cerebral palsy within the sample range one by one, without any omissions. Make sure that all the questionnaire items are filled in truthfully, and there are no missing items. In this study, a total of 55 questionnaires were distributed, and 55 valid questionnaires were returned. The effective response rate was 100%. After the on-site investigation, we reviewed the questionnaires, found problems, and resolved them in a timely manner. Researchers also conduct random surveys based on the telephone numbers or addresses of the respondents to ensure the quality of the questionnaire survey. In the entry part, the specially assigned persons entered and reviewed data to ensure that logging data was accurate.

The article "Investigation on Quality of Life and Economic Burden of Children with Cerebral Palsy in Changzhou" was retracted in 2023. Reasons: suspected computer-generated content; unreliable results or conclusions; concerns about the data; concerns about the results or conclusions.

## 3. Results

### 3.1. Demographic Characteristics of Children with Cerebral Palsy and Their Parents

Among the children with CP investigated, the youngest is 1 year old, the oldest is 13, and the average age is 5 years. Those under 10 years old accounted for 90.91% (50/55). Male children accounted for 70.91% (39/55), and females accounted for 29.09% (16/55).

The survey shows that 82% (45/55) of families live in cities. The average age of the mother is 33 years, and the father is 34. About 75% of parents have college, university, and above education level (father 41/55; mother 42/55). Most of their mothers were unemployed or private enterprise employees, accounting for 66.64% (35/55) of the total number, and most of their fathers were private enterprise employees or self-employed individuals, accounting for 74.55% (41/55) (Table 1).

### 3.2. Daily Activity Ability of Children with Cerebral Palsy

The vast majority of children with CP are poor in daily activities. Only 27.27% (15/55) of them can walk around, 20% (11/55) can take care of themselves, 18.18% (10/55) can perform daily activities, and 16.36% (9/55) do not have any pain or discomfort. Only 7.27% (4/55) of the children did not feel anxious or depressed (Table 2).

### 3.3. Direct Economic Burden of Children with Cerebral Palsy

Among the children with CP under investigation, 27.78% of them had comorbidities, and 9.62% had undergone surgery. 32.73% had been hospitalized in addition to surgery, and 65.45% of children had purchased rehabilitation equipment. 30.91% have purchased over-the-counter (OTC) drugs or nutritional products. 92.72% of them received rehabilitation treatment (Table 3).

According to the questionnaire conditions, 53 children should answer the source of medical expenses. The medical expenses of 68% of the children are sourced from social medical insurance and partially self-financed, and 22% are partially self-financed. Only 6% are completely self-financed, but only 4% completely come from social medical insurance (Figure 1).

The article "Investigation on Quality of Life and Economic Burden of Children with Cerebral Palsy in Changzhou" was retracted in 2023. Reasons: suspected computer-generated content; unreliable results or conclusions; concerns about the data; concerns about the results or conclusions.

The 33 children with cerebral palsy who had comorbidities without surgery or hospitalization were mainly due to mild symptoms (96.97%), followed by financial difficulties (3.03%).

Among the 55 valid questionnaires, we know that 100% of children with CP underwent general diagnosis and treatment, and their medical expenses averaged 15,900 yuan. Their accumulative total of transportation, accommodation, and escort expenses were 22,100 yuan. Twelve children (accounting for 21.82%) received surgical treatment, and their average medical expenses were 37,800 yuan, and the traffic, accommodation, and nursing fees added up to 71,600 yuan. There are 22 nonsurgical hospitalizations (accounting for 40%); the average was 35,800 yuan, and the addition of cost of transportation, accommodation, and accompany resulted a grand total of 44,800 yuan. Almost everyone chose rehabilitation treatment, the average medical cost was 105,900 yuan, and the cumulative total of others was 130,600 yuan. Among these expenses, the main one is medical expenses, followed by transportation costs, and the accommodation and escort costs are relatively low. Among the types of expenditures, the proportion of purchasing rehabilitation equipment for children is relatively high, and the proportion of purchasing nutritional products is relatively low (Table 4).

### 3.4. Indirect Economic Burden of Children with Cerebral Palsy

Among children with CP who cannot take care of themselves, the daily expenses of taking care of them cost an average of 5,500 yuan per month, and the total average family burden is about 293,500 yuan. In the survey, 11 children with CP received school education (including special kindergartens and auxiliary schools), accounting for 20%. The monthly special education fee is about 3,000 yuan, totaling 106,300 yuan (Table 5).

### 3.5. Economic Burden Calculation

Children with CP have different medical and family conditions. Not only are their treatment methods and types different, but also the utilization rate of various medical services is different. As a result, families actually bear different direct economic burdens. Children with serious comorbidities that require surgery, rehabilitation, and systemic treatment cost more. Those who are generally in better condition and have only undergone general diagnosis and treatment have relatively little medical expenses. In general, the direct economic burden of families with children ranges from 22,100 yuan to 285,600 yuan, with an average of 205,800 yuan.

According to the data released by Changzhou Municipal Government, in 2020, the urban per capita disposable income is 60,529 yuan, and the rural is 32,364 yuan [9]. It can be estimated that the actual indirect economic burden of each family is about 2.3006 million yuan for rural patients and about 4.3565 million yuan for urban patients, and the average is 3.9827 (2.306, 4.3565) million yuan. Affected by the income difference between rural residents and urban residents, the indirect burden of urban CP families is much higher than that of rural families. If patients with CP and their caregivers are transformed into normal labor, they will create value for society. Due to CP disease, this part of the production value is lacking, which constitutes the indirect economic burden of the society of this disease. According to the seventh census data [10], as of 0:00 on November 1, 2020, the permanent population of Changzhou is 5278121. In 2020, Changzhou achieved a regional gross product (GDP) of 780.53 billion yuan [9], so the per capita GDP is 147,800 yuan (Table 6).

The article "Investigation on Quality of Life and Economic Burden of Children with Cerebral Palsy in Changzhou" was retracted in 2023. Reasons: suspected computer-generated content; unreliable results or conclusions; concerns about the data; concerns about the results or conclusions.

To sum up, the economic burden of each family is 4.1885 (2.3227, 4.6421) million yuan. The actual social economic burden of 220 families with children with CP in Changzhou is about 2.244 billion yuan.

### 3.6. Quality of Life and Influencing Factors of Patients with Cerebral Palsy

The EQ-5D five-dimensional health status of patients with CP is not optimistic. The proportions of patients with CP who have moderate and severe problems in the five dimensions of action, self-care, daily activity ability, pain/discomfort, and anxiety/depression are 72.73%, 81.82%, 81.82%, 83.64%, and 92.73%, respectively (Table 7).

The average score of the 55 children with CP on the EQ-5D index was 0.423 (see Appendix 3).

The family life quality of patients with CP (VAS measurement data) is also low. In a total of 55 valid questionnaires, the average family score was 58.09, with the highest self-rating score of 90 and the lowest of 25. Only 19 patients scored 60 points or more, accounting for 34.55% of the total (Table 8).

We performed a grade correlation analysis on the EQ-5D index scores of children with CP and the family VAS scores and found that there was a significant correlation between the two (*R* = 0.811, *P* < 0.05). Those with a score less than 30 were regarded as the low quality of life group; otherwise, it was regarded as the high quality of life group. We first conduct a single-factor analysis of 13 factors and then include the meaningful variables (X7: *r* = −0.25422, *P*=0.0611; X9: *r* = 0.27527, *P*=0.0419; X13: *r* = 0.35902, *P*=0.0071) into logistic regression analysis (see Appendix 4). The stepwise logistic regression analysis showed that the only factor affecting the quality of family life of the children was the health status represented by the EQ-5D score (OR = 12.499 (1.338, 116.787)).

The article "Investigation on Quality of Life and Economic Burden of Children with Cerebral Palsy in Changzhou" was retracted in 2023. Reasons: suspected computer-generated content; unreliable results or conclusions; concerns about the data; concerns about the results or conclusions.

## 4. Discussion

According to calculations, the average family economic burden of each patient with cerebral palsy in Changzhou is about 4,188,500 yuan, of which the indirect economic burden accounts for the vast majority, and the direct medical burden accounts for only 4.91%. If calculated according to the average direct economic burden of each patient with CP, 193,500 yuan, it is 5.98 times as the per capita disposable income of rural residents in Changzhou in 2020 and 3.20 times as the per capita disposable income of urban residents. Meanwhile, owing to the fact that patients with CP and their caregivers are unable to engage in normal production all year round, their family income is low, which is generally lower than the average family income. Moreover, they seldom participate in social production and create labor value, which leads to a significantly larger indirect economic burden on society. In the light of the human capital method, the socioeconomic burden of 220 children with CP in Changzhou is as high as 2.244 billion yuan, accounting for 0.29% of Changzhou's GDP in 2020.

The data on direct family medical costs of patients with CP is distributed skewedly and varies greatly. This is mainly related to service utilization, family economic status, urban-rural differences, and social security. Our investigation found that the utilization rate of general diagnosis and rehabilitation treatment is very high, but the rate of purchasing nutritional products and rehabilitation equipment is low. Moreover, rural patients' access to related services is significantly harder than that of urban patients. Most of these patients with CP have a poor prognosis and usually fall into a vicious circle where the less the money they have for treatment, the worse their health and self-care ability and the heavier the indirect burden. Social security will reduce the financial burden of patients' families to a certain extent, but it is difficult to achieve full coverage.

Our further analysis found that the main factors affecting the social and economic burden are the incidence of disease and the rate of recovery. Obviously, reducing the incidence of diseases can directly reduce the number of patients with CP, thereby reducing the socioeconomic burden. Increasing the recovery rate means liberating and developing the labor force, and it can also fundamentally reduce the indirect economic burden. Due to motor dysfunction, children with cerebral palsy often have changes in their psychology and mental state, and it is difficult to adapt to society. Therefore, special education must be carried out to correctly understand themselves, build confidence, and eliminate man-made bad psychological factors. As long as they are given the help they deserve, children with cerebral palsy can become talents and contribute to society. Without special education, other rehabilitation works will be difficult to carry out. Therefore, on the whole, interventions and funding of social and government should mainly focus on three aspects: early clinical treatment, standardized rehabilitation, and science education for patients with CP.

The article "Investigation on Quality of Life and Economic Burden of Children with Cerebral Palsy in Changzhou" was retracted in 2023. Reasons: suspected computer-generated content; unreliable results or conclusions; concerns about the data; concerns about the results or conclusions.

Through family interviews, we also learned about the invisible burden of CP patients and their families. Because of communication problems in patients with CP, most of our interviews were with their parents or direct caregivers. In the interview, almost all the interviewees believed that CP disease not only brought heavy economic pressure to the family but also overwhelmed the invisible burdens such as social discrimination, psychological load, and family problems. Many family members expressed pain, helplessness, grief, and despair.

From EQ-5D measurement results, the proportions of patients with CP who have problems in five aspects, namely, action, self-care, daily activity ability, pain/discomfort, and anxiety/depression, are 72.73%, 81.82%, 81.82%, 83.64%, and 92.73%, respectively. The average EQ-5D score of 55 children with CP in Changzhou is 0.423. According to the EQ-5D scale survey for 2994 urban residents in Beijing, the proportions of problems in the five aspects are 3.4%, 1.4%, 2.2%, 13.0%, and 5.3%, respectively. The average score of their EQ-5D index is 0.77 [11]. The proportions from 2830 rural residents in Kaiyang County, Guizhou Province, are 5.95%, 3.39%, 8.19%, 25.03%, and 33.23%, and the average EQ-5D score is 0.67 [12]. The proportions of the five aspects of children with CP in Hebei Province are 87.81%, 94.34%, 94.34%, 58.43%, and 72.05%, and the average score of the EQ-5D index is 0.44 [8]. By comparison, we find that the proportion of children with CP in Changzhou who have problems in the five dimensions is significantly higher than that of the general population, and the average score of the EQ-5D index is significantly lower than that of the general population. Our results are similar to those of the children with CP in Hebei Province.

We asked the direct caregivers to score themselves based on the current quality of life. The average score is 58.09, and there are 19 people with a score of 60 or more, accounting for 34.55% of the total. This result is significantly higher than that in Hebei Province [8]. The average VAS score of children in Hebei Province is 27, 50% of which scored below 30, and those with a score of 60 or above accounted for only 5.9% of the total.

The article "Investigation on Quality of Life and Economic Burden of Children with Cerebral Palsy in Changzhou" was retracted in 2023. Reasons: suspected computer-generated content; unreliable results or conclusions; concerns about the data; concerns about the results or conclusions.

With reference to VAS scores of the health-related quality of life of the general population, the fourth health service survey in China in 2008 [13] showed that the VAS scores of the general population in rural areas was 80.4. Comparing the VAS score, we found that the VAS score of patients with CP and their families in Changzhou is lower than that of the general population but higher than that in Hebei Province [8]. Parents of most families who take care of children with cerebral palsy often have mental and physical disorders such as perseverance and sensitivity and may be accompanied by emotional problems such as autism, depression, and anxiety. These health problems and negative emotions make them show strong dissatisfaction with the status quo of the family. Well-being is thus reflected in the low scores of VAS. Similarly, the quality of life of parents of patients with CP has also significantly decreased [14–16]. Through stepwise logistic regression analysis, we found that the only factor affecting the quality of life of the children's family was the EQ-5D score. Domestic research in Hebei Province shows that EQ-5D score, hospitalization, surgical treatment, mother's education level, presence of brothers and sisters, and school education are the influencing factors. Schneider's research has shown [17] that parental care time, family cohesion, and the ability to receive school education significantly affect the quality of life of children with CP. Our conclusions are similar to and different from those of domestic and foreign research. The different conclusions may be that our sample size needs to be further expanded.

In recent years, the news media has repeatedly reported on cases of CP patients and family plights. The misfortune of CP patients' families has attracted more and more social attention. However, due to the lack of basic data on cerebral palsy, most people believe that the incidence of this disease is low and the disease burden is limited, especially since it has not received high attention and policy support from relevant government departments. From an empirical point of view, this study demonstrates that not only does cerebral palsy restrict family development but also the economic burden of the disease is quite alarming. At the same time, from a social perspective, cerebral palsy can also lead to social problems such as abandonment of infants and family breakdown. Therefore, relevant government departments should attach great importance to the major harm of cerebral palsy and take active and effective countermeasures.

Although the demographic characteristics, sociological characteristics, and health conditions of our respondents and the participants of other groups are not very homogeneous, such intuitive comparison may not be able to directly draw an authoritative conclusion, but the serious impact of CP on the quality of life of patients and their families is obvious. Some treatments and interventions have been shown to be cost-effective, although stronger evidence of clinical effectiveness is needed [18].

The article "Investigation on Quality of Life and Economic Burden of Children with Cerebral Palsy in Changzhou" was retracted in 2023. Reasons: suspected computer-generated content; unreliable results or conclusions; concerns about the data; concerns about the results or conclusions.

## 5. Conclusion

This paper adopts a quantitative analysis method to calculate the present situation of the family and socioeconomic burden of cerebral palsy in Changzhou. The calculated data intuitively reflects that the economic burden caused by cerebral palsy is very heavy. At the same time, a comprehensive evaluation of the quality of life of children with cerebral palsy and their families was carried out by using the EQ-5D scale, which objectively reflects that cerebral palsy has seriously affected the quality of life, family happiness, and social harmony. We found that to liberate and develop the labor capacity of patients and their direct caregivers through clinical treatment, rehabilitation, and special education is the most effective way to reduce the socioeconomic burden of cerebral palsy and improve the quality of life. This study is conducive to government departments and social community to fully understand the great harm of cerebral palsy and the necessity and urgency of intervention measures.

## Figures and Tables

**Figure 1:** Sources of medical expenses for children with cerebral palsy.

**Table 1:** Demographic characteristics of parents of children with cerebral palsy.

		Mother (*n*, %)	Father (*n*, %)
Age		33.24 ± 4.20	34.18 ± 4.45
Profession	Unemployed	18 (35.73)	1 (1.82)
	Self-employed	3 (5.45)	8 (14.55)
	Employees of government agencies	12 (21.82)	5 (9.09)
	Migrant workers	1 (1.82)	1 (1.82)
	Others	3 (5.45)	1 (1.82)
	Employees of private enterprises	17 (30.91)	33 (60.00)
	Professional technicians	1 (1.82)	6 (10.91)
Degree of education	Illiterate or semi-illiterate	0 (0.00)	0 (0.00)
	Primary school and below	0 (0.00)	0 (0.00)
	Junior middle school	6 (10.91)	5 (9.09)
	High school, vocational school, and technical secondary school	7 (12.73)	9 (16.36)
	College, university, or above	42 (76.36)	41 (74.55)

**Table 2:** Daily activity ability of children with cerebral palsy.

		Number of people	Proportion (%)
**D1** action	I can walk around without any difficulty	15	27.27
	It is a little inconvenient for me to move	26	47.27
	I cannot get out of bed and move around	14	25.45
**D2** self-care	I can take care of myself without any difficulties	11	20.00
	I have some difficulties in washing my face, brushing my teeth, bathing, or getting dressed	26	47.27
	I cannot wash my face, brush my teeth, bathe, or dress myself	19	34.55
**D3** daily activities (such as work, study, housework, family, or leisure activities)	I can carry out daily activities without any difficulties	10	18.18
	I have some difficulties in carrying out daily activities	29	52.73
	I cannot carry out daily activities	16	29.09
**D4** pain or discomfort	I do not have any pain or discomfort	9	16.36
	I feel moderately pain or discomfort	33	60.00
	I feel extremely painful or uncomfortable	13	23.64
**D5** anxiety (such as nervousness, worry, anxiety, etc.)/depression (such as lack of interest in doing things, no fun, lack of energy, etc.)	I do not feel anxious or depressed	4	7.27
	I feel moderately anxious or depressed	36	65.45
	I feel extremely anxious or depressed	15	27.27

The article "Investigation on Quality of Life and Economic Burden of Children with Cerebral Palsy in Changzhou" was retracted in 2023. Reasons: suspected computer-generated content; unreliable results or conclusions; concerns about the data; concerns about the results or conclusions.

**Table 3:** Treatment of children with cerebral palsy.

	Number of people who should be answered	Answer “yes” (*n*, %)
Whether there are comorbidities	54	15 (27.78)
Whether to undergo surgery	52	5 (9.62)
In addition to surgery, whether to be hospitalized	55	18 (32.73)
Whether to buy rehabilitation equipment	55	36 (65.45)
Whether to take over-the-counter drugs or nutritional products	55	17 (30.91)
Whether to receive rehabilitation	55	51 (92.73)

**Table 4:** Relevant treatment costs for children with cerebral palsy (unit: ten thousand yuan).

	Number of people	Medical expense	Transportation expense	Accommodation expense	Escort expense	Total
General diagnosis and treatment expenses	55	0.50 (0.20, 2.00)	0.23 (0.03, 0.2)	0.03 (0, 0.2)	0.27 (0.13, 0.65)	1.56 (0.46, 4.58)
Surgical treatment expenses	12	3.00 (3.00, 5.25)	0.06 (0.05, 0.50)	0.3 (0, 0.46)	0.25 (0.20, 0.54)	3.74 (1.65, 6.99)
Nonsurgical hospitalization expenses	22	2.5 (1.00, 5.00)	0.10 (0.05, 0.175)	0.3 (0.00, 0.3)	0.49 (0.33, 0.61)	3.56 (0.61, 6.53)
Rehabilitation treatment expense	55	7.20 (5.00, 7.20)	0.50 (0.24, 1.00)	2.00 (0.50, 7.00)	0.35 (0.00, 0.40)	11.03 (5.12, 9.55)
The cost of purchasing supplements	18	0.4 (3, 0.97)	—	—	—	0.4 (0.13, 0.97)
The cost of purchasing rehabilitation equipment	36	0.29 (18, 0.56)	—	—	—	0.29 (0.18, 0.56)

**Table 5:** Indirect economic burden of children with cerebral palsy.

	Number of people	Time (month)	Average monthly cost (ten thousand yuan)	Total cost (ten thousand yuan)
Daily care expenses	12	47.70 (5.28, 67.65)	0.55 (38, 0.6)	29.35 (5.64, 38.47)
Special education expenses	11	42.00 (6.00, 62.00)	0.30 (14, 0.35)	10.63 (56, 19.68)

**Table 6:** Calculation table of actual indirect family burden and social indirect burden of children with cerebral palsy.

	Time (year)	Per capita annual income (ten thousand yuan)		GDP per capita (ten thousand yuan)	Number of children or caregivers		Total social indirect burden (ten thousand yuan)
		Urban	Rural		Urban	Rural	
Patient labor	42	6.0529	3.2364	14.788	45	10	34160.28
Direct caregiver labor	27	6.0529	3.2364	14.788	45	10	21960.18
Special education	9	−1	−0.75	—	11	0	—
The actual indirect burden of each family	—	435.65	230.06	—	—	—	56120.46

The article "Investigation on Quality of Life and Economic Burden of Children with Cerebral Palsy in Changzhou" was retracted in 2023. Reasons: suspected computer-generated content; unreliable results or conclusions; concerns about the data; concerns about the results or conclusions.

**Table 7:** EQ-5D five-dimensional health status of children with cerebral palsy.

Total number of valid questionnaires	No problem		Moderate problems		Severe problems	
	Number of people	Composition ratio (%)	Number of people	Composition ratio (%)	Number of people	Composition ratio (%)
55	15	27.27	26	47.27	14	25.45
55	11	20.00	26	47.27	19	34.55
55	10	18.18	29	52.73	16	29.09
55	9	16.36	33	60.00	13	23.64
55	4	7.27	36	65.45	15	27.27

**Table 8:** Visual Analogue Scale of children with cerebral palsy.

Score	Number of people	Percentage	Cumulative percentage
0∼10	0	0	0
∼20	0	0	0
∼30	5	9.09	9.09
∼40	11	20	29.09
∼50	12	21.82	50.91
∼60	8	14.55	65.46
∼70	5	9.09	74.55
∼80	10	18.18	92.73
∼90	4	7.27	100
∼100	0	0	100
Total	55	100	100

## Data Availability

The data in this study are all derived from questionnaire surveys. As it involves the privacy of cerebral palsy patients and their direct caregivers, the data cannot be fully disclosed. If the research colleagues are interested in this, you can contact the corresponding author via email to obtain the data.

## Supplementary Materials

Supplementary Materials Appendix 1: the informed consent form and the questionnaire used in this survey. Appendix 2: the detailed introduction of the calculation method of economic burden and the EQ-5D scale. Appendix 3: the EQ-5D index of 55 children with cerebral palsy. Appendix 4: the specific assignment of a dependent variable and 13 independent variables.
